The article "Long Noncoding RNA LOC554202 Predicts a Poor Prognosis and Correlates with Immune Infiltration in Thyroid Cancer" was published in 2022. Journal: Comput Math Methods Med.

# Long Noncoding RNA LOC554202 Predicts a Poor Prognosis and Correlates with Immune Infiltration in Thyroid Cancer

**DOI:** 10.1155/2022/3585626

**Published:** 2022-02-28

**Authors:** Cheng Chen, Lu Qin, Mei-Fang Xiao

**Affiliations:** ^1^Department of Nuclear Medicine, Jingzhou Central Hospital, Jingzhou, Hubei 434020, China; ^2^Department of Thyroid Vascular Surgery, Jingzhou Central Hospital, Jingzhou, Hubei 434020, China; ^3^Center for Laboratory Medicine, Hainan Women and Children's Medical Center, Haikou, Hainan 570206, China

## Abstract

Thyroid cancer (TC) is one of the widely diagnosed carcinomas in women before the age of 30. Nevertheless, there is currently a lack of specific biomarkers for predicting the prognosis of TC. Long noncoding RNAs (lncRNAs) were important regulators in human cancer progression as previously described. Unfortunately, there is little known on these lncRNAs' functions and molecular mechanisms in TC. In our literature, we found that LOC554202 (MIR31HG) was upregulated in TC samples and correlated with clinicopathological features, including M stage, N stage, and lymph nodes examined status in TC. In addition, we found that LOC554202 overexpression was evidently correlated with high immune infiltrate levels of CD8+ T cells, macrophage, neutrophil, myeloid dendritic cells, and B cells in TC. Knockdown of LOC554202 impeded TC cell proliferation and cycle progression. We found that LOC554202 had an association with metabolic pathways, vesicle-mediated transport, tricarboxylic acid cycle, Hedgehog signaling pathway, and Hippo signaling pathway in TC. Reducing LOC554202 hindered TC cell proliferation and cycle progression. Finally, we found that LOC554202 participated in modulating the expression of the regulators of Hippo signaling and TCA pathway, such as CCND2, CCND3, SDHC, SDHD, SUCLA2, and SUCLG1. We thought that this study would largely enhance our understanding of LOC554202's functional roles in human TC progression and immune response.

## 1. Introduction

Thyroid cancer (TC) is one of the widely diagnosed carcinomas in women before the age of 30. Nevertheless, there is currently a lack of specific biomarkers for predicting the prognosis of TC. Long noncoding RNAs (lncRNAs) are endogenous RNA transcripts with a length of more than 200 nucleotides. It has shown that lncRNAs function as an important modulator of human carcinoma progression. lncRNAs played oncogenic or tumor suppressive roles via modulating several biological processes, including cell proliferation, metastasis, and epithelial-mesenchymal transition. lncRNAs played their roles through interacting with other cellular macromolecules including DNA, RNA, and proteins. Several groups investigated the roles of lncRNAs in TC tumorigenesis and progression. For example, Xu et al. reported that ENST00000537266 and ENST00000426615 could inhibit cell proliferation in TC [1]. Nonetheless, it was not well understood on most of lncRNAs' functions and molecular mechanisms in TC.

The lncRNA LOC554202 was firstly reported to be upregulated in breast cancer. Higher expression of LOC554202 exhibited an association with advanced pathologic stage and tumor size in breast carcinoma [2]. LOC554202 expression was also found to be overexpressed in laryngeal squamous cell carcinoma, oral cancer, and lung adenocarcinoma [3–6]. Interestingly, several groups identified that LOC554202 was downregulated in bladder carcinoma and gastric carcinoma [7, 8]. Previous studies demonstrated that LOC554202 participated in the regulation of gefitinib resistance, cell proliferation, and migration [9–11]. These findings further implied that LOC554202 was a potential biomarker for human carcinomas. Nevertheless, it was not well documented regarding the expression pattern and potential molecular functions of LOC554202 in TC.

In the present study, we analyzed the LOC554202 expression pattern in TC by analyzing public datasets. The influence of LOC554202 on cell proliferation and cell cycle was evaluated by loss of function assays. Our findings collectively provided useful information to support that LOC554202 could be a novel biomarker for TC.

## 2. Materials and Methods

### 2.1. Public Dataset Analysis

LOC554202 expression levels in thyroid cancer (TC) were analyzed by TCGA and GSE50901 [12] datasets. GSE50901 was uploaded by Barros-Filho MC which consists of 57 PTC with a reference sample (pool of 9 adjacent normal thyroid tissue) and 4 PTC against 4 matched adjacent normal thyroid tissues. The clinical information of LOC554202 was obtained from cBioPortal [13, 14] (http://www.cbioportal.org/). The stage of patients was evaluated by 2009 Tumor-Node-Metastasis (TNM) classification.

### 2.2. GO and KEGG Pathway Analysis

The Pearson correlation coefficient of the LOC554202-gene pair was calculated. The coexpressed LOC554202-mRNA pair with an absolute Pearson correlation coefficient ≥ 0.3 was chosen for analysis. GO and KEGG pathway analysis was employed for predicting LOC554202's biological function using the MAS3.0 system (http://bioinfo.capitalbio.com/mas3/). The *p* value < 0.05 meant there was a significant statistical difference.

### 2.3. Cell Culture and Transfection

CAL62 and SW579 cells were acquired from the American Type Culture Collection. Both of them were cultured in L-15 medium containing 10% FBS (GIBCO) under a 37°C incubator with 5% CO_2_. siRNA for LOC554202 (5′-CCUGGUUGAGCUGAGGUCUUCAUAG-3′) and siNC was purchased from RiboBio. Transfection was performed using Lipofectamine 3000.

### 2.4. Real-Time Reverse Transcription PCR (qRT-PCR) Analysis

Overall RNAs were harvested with the use of the Ultrapure RNA Kit (CWBIO, China). And reverse transcription of RNA was performed with the PCR PrimeScript™ RT reagent kit (TaKaRA, China). The gene expression values were derived from the Ct values which were normalized to internal control *β*-actin. The 2-*ΔΔ*Ct method was used to calculate the relative mRNA expression. All data were obtained from three separate experiments in triplicate.

### 2.5. Cell Proliferation and Cycle Assay

We used CCK-8 assays to detect cell proliferation after transfection. 100 *μ*l medium/well of transfected cells was plated in a 96-well plate at the appropriate density. Proliferation was detected at 0 d, 1 d, 2 d, 3 d, and 4 d. 10 *μ*l medium/well of CCK-8 (Dojindo, Japan) was added before detection, then incubation for 1.5 hours; the absorbance at 450 nm was measured by a microplate reader. The absorbance wavelength at 630 nm was an internal reference. Regarding cell cycle detection, all indicated cells were collected and incubated with the indicated concentration of triton X-100 and propidium iodide (PI) for 20 min, followed by observation with a flow cytometer (Beckman, USA).

### 2.6. Statistical Analysis

In the light of the test condition, the *T*-test or Mann–Whitney *U*-test was utilized for statistical comparisons in two groups. One-way ANOVA followed by the Newman-Keuls post hoc test was used for multiple comparisons in several groups. The association of LOC554202 expression with disease-free survival (DFS) and the prognosis of prostate cancer was analyzed by Kaplan-Meier and Cox regression analyses. A *p* value < 0.05 was considered statistically significant. The SPSS 15.0 software package (SPSS Inc., Chicago, IL) was applied for data analysis.

## 3. Results

### 3.1. lncRNA LOC554202 Was Overexpressed in TC

We analyzed TCGA dataset to evaluate the expression pattern of LOC554202 in TC. We found that higher expression of LOC554202 was in TC tissues rather than that in the normal samples by analyzing GSE50901 (Figure 1(a)) and TCGA (Figure 1(b)). Furthermore, we determined LOC554202 levels in 58 paired TC samples in TCGA data. Among these pair samples, 80 percent of cases (51/58) displayed higher levels of LOC554202 in PTC samples in comparison with that in adjacent normal samples (Figures 1(c) and 1(d)).

### 3.2. Higher LOC554202 Expression Was Correlated with Clinicopathological Characteristics in TC

We in-depth assessed the correlations of LOC554202 expression with clinicopathological traits in TC. As shown in Figure 2, we found that LOC554202 was overexpressed in M0 compared to M1 and Mx (Figure 2(a)), in N1 and Nx stage TC compared to N0 stage samples (Figure 2(b)), and in lymph nodes examined positive compared to lymph nodes examined negative samples (Figure 2(c)). However, we did not find the LOC554202 expression correlated with T stage, residual tumor status, age, and gender. Our data reflected that LOC554202 was a promising biomarker for TC.

### 3.3. Higher LOC554202 Expression Was Correlated with Higher Levels of Immune Infiltration in TC

The correlation between LOC554202 expression and immune infiltration levels was detected using the TIMER database. The TC samples were divided into the LOC554202-high and LOC554202-low groups based on the median expression of LOC554202. As presented in Figure 3, we found that CD8+ T cells, macrophage, neutrophil, myeloid dendritic cells, and B cell levels were higher in LOC554202-high TC samples than that in LOC554202-low TC samples (Figures 3(a) and 3(b)). Moreover, the correlation analysis demonstrated that higher LOC554202 expression was correlated with higher levels of immune infiltration of CD8+ T cells, macrophage, neutrophil, myeloid dendritic cells, CD4+ T cells, and B cell levels in TC by analyzing the TIMER database (Figures 4(a)–4(f)).

### 3.4. Bioinformatics Analysis of LOC554202 in TC

Coexpression analysis and functional analysis including GO and KEGG pathway were used to investigate LOC554202's function in TC. We totally identified 1385 of LOC554202-mRNA pairs according to the cutoff which meant the absolute value of Pearson correlation coefficient ≥ 0.30.

Furthermore, we utilized the DAVID system to forecast LOC55420's potential functions in TC. Our data indicated that LOC554202 had an association with branched-chain amino acid catabolic process, coronary vasculature development, neuron projection morphogenesis, ER to Golgi vesicle-mediated transport, tricarboxylic acid cycle, vesicle-mediated transport, peptidyl-serine phosphorylation, neural tube closure, protein phosphorylation, negative regulation of GTPase activity, protein binding, electron carrier activity, calcium-dependent phospholipid binding, fatty-acyl-CoA binding, SH3 domain binding, ATP binding, kinase activity, thiamine pyrophosphate binding, acyl-CoA dehydrogenase activity, and protein serine/threonine kinase activity (Figures 5(a) and 5(b)).

KEGG pathway analysis revealed that LOC554202 participated in regulating metabolic pathways, Hedgehog signaling pathway, Hippo signaling pathway, adipocytokine signaling pathway, RIG-I-like receptor signaling pathway, and sphingolipid signaling pathway (Figure 5(c)).

### 3.5. Knockdown of LOC554202 Inhibited Cell Proliferation and Cell Cycle in TC

For evaluating LOC554202's roles in TC, we carried out the CCK-8 assay and flow cytometer analysis. We discovered that compared to the normal control cells, LOC554202 was greatly downregulated in cells with ablated LOC554202. Besides, we found that compared to the normal control cells, TC cell proliferation at 72 h was inhibited upon silencing LOC554202 (Figures 6(a) and 6(b)). The cell cycle assay indicated that reduced LOC554202 in TC cells mediated cell cycle modulation through arresting G0/G1. Enhanced LOC554202 led to the increase in the ratio of S stage but the decrease in the ratio of G0/G1 phase in TC cells (*p* < 0.01, Figures 6(c)–6(f)).

### 3.6. Knockdown of LOC554202 Suppressed CCND2 and CCND3 Expression in Thyroid Cancer

KEGG pathway analysis presented that LOC554202 took part in the regulation of Hippo signaling in TC. As shown in Figure 5, we found LOC554202 positively coexpressed with 14 genes in Hippo signaling, including BBC3, GLI2, SMAD2, TEAD3, WNT10A, BMP4, BMP7, CSNK1E, CRB1, CCND2, CCND3, DLG2, DLG4, DVL1, GDF6, ID2, LATS2, TCF7L2, and TGFB1. Among these genes, we focused on CCND2 and CCND3, which were cell cycle regulators and involved in promoting cell proliferation in cancer cells. CCND2 and CCND2 expression levels were positively coexpressed with LOC554202 in TCGA dataset (Figures 7(a) and 7(c)). CCND2 and CCND2 expression levels were furthermore detected in TC cells with LOC554202 knockdown by RT-PCR. Our results showed that CCND2 and CCND2 expression in mRNA levels were obviously suppressed after LOC554202 knockdown in TC cells (Figure 7(b)).

### 3.7. Knockdown of LOC554202 Induced Tricarboxylic Acid Cycle Regulator Expression in Thyroid Cancer

Very interestingly, we found that LOC554202 expression levels in TC samples were significantly negatively correlated with the gene expression of tricarboxylic acid cycle regulators, suggesting that LOC554202 may suppress tricarboxylic acid cycle progression in TC. Therefore, we explored the impacts of LOC554202 on tricarboxylic acid cycle regulators, including DHTKD1, DLAT, OGDH, OGDHL, SDHC, SDHD, SUCLA2, SUCLG2, and SUCLG1 (Figures 8(a)–8(i)). RT-PCR detection displayed that LOC554202 knockdown greatly promoted the levels of DLAT, OGDH, OGDHL, SDHC, SDHD, SUCLA2, and SUCLG1, suggesting that LOC554202 may be involved in suppressing the TCA process in TC (Figure 8(j)).

## 4. Discussion

Previous studies had reported that lncRNAs exerted their tissue specificity in various carcinomas and exhibited importantly in tumorigenesis and progression. lncRNA OCC-1 was shown to mediate the suppression of cell growth via destabilizing HuR in colorectal carcinoma [15]. FEZF1-AS1 could regulate PKM2 signaling, thus promoting cell proliferation and metastasis in colorectal carcinoma [16]. lncRNA MIR4435-2HG was found to promote the progression of lung cancer via activating *β*-catenin signaling [17]. TC is a common endocrine malignancy in women, whose incidence is increasing in the past decade. Several lncRNAs, including TNRC6C-AS [18], AFAP1-AS1 [19], GAS8-AS1 [20], NONHSAT129183 [21], and MALAT1 [22], were found to be associated with tumor progression in TC. Nevertheless, it was still elusive towards the role of LOC554202 in TC. Our study suggested that lncRNA LOC554202 was overexpressed in TC samples compared to normal ones. Furthermore, LOC554202 expression in our research displayed a correlation with clinicopathological features, including M stage, N stage, and lymph nodes examined status in TC. Our study for the first time presented that higher expression of LOC554202 had a correlation with higher levels of immune infiltration in TC. We also for the first time uncovered that LOC554202 functioned as a novel biomarker for predicting the immune cell infiltration levels and prognosis of TC.

Previous studies had showed that the tumor microenvironment participated in modulating tumor initiation, progression, and immune therapy response in human cancers. Higher expression of CD4+ T cells and CD8+ T cells was observed in TC samples. Of note, this study for the first time revealed that LOC554202 overexpression significantly correlates with high infiltrate levels of multiple immune cells, such as CD8+ T cells, macrophage, neutrophil, myeloid dendritic cells, and B cells in TC.

In the past few years, LOC554202 was found to be dysregulated in human cancers and showed potential prognostic values in predicting cancer outcomes. LOC554202 was found to be overexpressed in laryngeal squamous cell carcinoma, oral cancer, and lung adenocarcinoma and downregulated in bladder carcinoma, gastric carcinoma, colorectal carcinoma, and esophageal squamous cell carcinoma [3–6]. LOC554202 regulated cancer progression by influencing various types of human cancers, including proliferation, migration, apoptosis, invasion, and hypoxia response. Shih et al. found that LOC554202 was a hypoxia-inducible lncRNA and regulates the HIF-1 transcriptional network to promote oral cancer progression through interacting with HIF-1*α* [4]. In pancreatic ductal adenocarcinoma, ablating MIR31HG largely hindered cell growth and cell invasion of PDAC but induced cell apoptosis and G1/S arrest [23]. In this study, we performed the loss of function assay and observed that silencing of LOC554202 significantly suppressed TC cell proliferation and arrested cell cycle in G0/G1 stage. This study showed that LOC554202 functioned as an oncogene in TC.

Coexpression analysis was the largely applied method to uncover lncRNAs' roles. In this study, we combined coexpression analysis and GO and KEGG pathway analysis to reveal molecular functions of LOC554202 in TC. The present study showed LOC554202 significantly involved in regulating metabolic pathways, tricarboxylic acid cycle, Hedgehog signaling pathway, Hippo signaling pathway, adipocytokine signaling pathway, RIG-I-like receptor signaling pathway, and sphingolipid signaling pathway. Of note, we found LOC554202 positively coexpressed with 14 genes in Hippo signaling, including BBC3, GLI2, SMAD2, TEAD3, WNT10A, BMP4, BMP7, CSNK1E, CRB1, CCND2, CCND3, DLG2, DLG4, DVL1, GDF6, ID2, LATS2, TCF7L2, and TGFB1. Hippo signaling played an important role in cancer growth, apoptosis, and development. CCND2 and CCND3 were cell cycle regulators. Previous studies had demonstrated that CCND2 acted as an oncogene in TC cells. Our literature revealed that LOC554202 knockdown greatly suppressed both CCND2 and CCND3 mRNA and protein levels in TC cells. These results suggested that LOC554202 promoted TC proliferation and cell cycle through upregulating CCND2 and CCND3.

Glycolysis was a hallmark of cancer cells. As we all know, cancer cells preferred to produce energy through the glycolysis pathway. The upregulation of glycolysis was observed in multiple human cancers. However, the mechanism underlying the downregulation of TCA needed to be further addressed. In our research, we found that LOC554202 expression had a negative correlation with the TCA regulators. Knockdown of LOC554202 remarkably promoted the expression levels of DLAT, OGDH, OGDHL, SDHC, SDHD, SUCLA2, and SUCLG1. These results suggested that LOC554202 may suppress the TCA process in TC and serve as a switch to turn off the TCA process.

We also noted several limitations in this study. First, the expression pattern of LOC554202 in cancers was analyzed using TCGA and GSE50901 datasets. Further confirmation of the LOC554202 expression in thyroid cancer using clinical samples is still needed. Second, the effects of LOC554202 on cell proliferation were confirmed using the CCK-8 kit. More confirmation such as the cell cycle assay and cell apoptosis assay is needed. Third, bioinformatics analysis showed that LOC554202 was related to modulating Hippo and TCA signaling and affects the tumor immune infiltration. However, the detailed mechanisms require to be further explored.

## 5. Conclusions

In summary, our current data revealed that LOC554202 was enhanced in TC samples and was correlated with clinicopathological features, including M stage, N stage, and lymph nodes examined status in thyroid cancer. Moreover, we revealed that LOC554202 overexpression significantly correlates with high immune infiltrate levels of CD8+ T cells, macrophage, neutrophil, myeloid dendritic cells, and B cells in TC. Bioinformatics analysis showed that LOC554202 was linked to metabolic pathways, vesicle-mediated transport, protein phosphorylation, tricarboxylic acid cycle, Hedgehog signaling pathway, and Hippo signaling pathway in TC. Reducing LOC554202 hindered TC cell proliferation and cycle progression. Finally, we found that LOC554202 participated in modulating the expression of the regulators of Hippo signaling and TCA pathway. Our study would largely enhance our understanding of the functional roles of LOC554202 in human TC progression.

## Figures and Tables

**Figure 1:** LOC554202 was upregulated in TC. In GSE50901 (a) and TCGA (b) datasets, LOC554202 expression was enhanced in TC compared to normal samples. (c, d) LOC554202 was upregulated in PTC samples compared to the adjacent normal samples (^∗∗∗^*p* < 0.001).

**Figure 2:** Higher LOC554202 expression was associated with clinicopathological characteristics in TC. LOC554202 was overexpressed in M0 compared to M1 and Mx (a), in N1 and Nx stage TC compared to N0 stage samples (b), and in lymph nodes examined positive compared to lymph nodes examined negative samples (c). (e, f) LOC554202 expression was not correlated with the T stage, residual tumor status, age, and gender (^∗∗^*p* < 0.01; ^∗∗∗^*p* < 0.001).

**Figure 3:** Higher LOC554202 expression was positively correlated with higher levels of immune infiltration in TC. (a, b) The CD8+ T cells, macrophage, neutrophil, myeloid dendritic cells, and B cell levels were higher in LOC554202-high TC samples than that in LOC554202-low TC samples.

**Figure 4:** The higher LOC554202 expression was positively correlated with higher levels of immune infiltration of B cell levels (a), CD4+ T cells (b), CD8+ T cells (c), neutrophil (d), macrophage (e), and myeloid dendritic cells (f) in TC by analyzing TIMER database.

**Figure 5:** Bioinformatics analysis of LOC554202 in TC. GO (a), molecular function (b), and KEGG (c) pathway analysis for LOC554202 in TC by using its coexpressing genes.

**Figure 6:** The knockdown of LOC554202 inhibited cell proliferation in TC. The knockdown of LOC554202 significantly suppressed TC cell proliferation at 72 h (a, b). The knockdown of LOC554202 in TC cells inhibited the cell cycle (c, d) (^∗∗^*p* < 0.01; ^∗∗∗^*p* < 0.001).

**Figure 7:** Knockdown of LOC554202 suppressed CCND2 and CCND3 expression in thyroid cancer. (a, c) The CCND2 and CCND2 expression levels were positively correlated with higher LOC554202 expression. The CCND2 and CCND3 expression in mRNA (b) was obviously suppressed after LOC554202 knockdown in TC cells.

**Figure 8:** Knockdown of LOC554202 induced tricarboxylic acid cycle regulator expression in TC. LOC554202 expression levels were significantly negatively correlated with the gene expression of tricarboxylic acid cycle regulators in TCGA dataset, including DLAT, DHTKD1, SDHC, SDHD (d), OGDH, SUCLA2, SUCLG1, OGDHL, and SUCLG2. (b) Knockdown of LOC554202 promoted the mRNA expression levels of DLAT, OGDH, OGDHL, SDHC, SDHD, SUCLA2, and SUCLG1 in TC.

## Data Availability

Previously reported lncRNA data were used to support this study and are available at doi:10.1210/jc.2014-4053. These datasets are cited at relevant places within the text as references [12].
